The article "Prediction of Incidence Trend of Influenza-Like Illness in Wuhan Based on ARIMA Model" was retracted in 2023. Reasons: signs of a paper mill; suspected computer-generated content; unreliable results or conclusions; lack of ethics approval or compliance.

# Prediction of Incidence Trend of Influenza-Like Illness in Wuhan Based on ARIMA Model

**DOI:** 10.1155/2022/6322350

**Published:** 2022-07-12

**Authors:** Pai Meng, Juan Huang, Deguang Kong

**Affiliations:** Wuhan Center for Disease Prevention and Control, Wuhan, China

## Abstract

**Objective:**

The autoregressive integrated moving average (ARIMA) model has been widely used to predict the trend of infectious diseases. This paper is aimed at analyzing the application of the ARIMA model in the prediction of the incidence trend of influenza-like illness (ILI) in Wuhan and providing a scientific basis for the prediction and prevention of influenza.

**Methods:**

The weekly ILI data of two influenza surveillance sentinel hospitals in Wuhan City published on the website of the National Influenza Center of China were collected, and the ARIMA model was used to model the data from 2014 to 2020, to predict and verify the ILI data in 2021.

**Results:**

The optimal model for the incidence trend of ILI in Wuhan was ARIMA (1, 1, 1), the residuals were in line with the white noise sequence (0.018 < Ljung‐Box *Q* < 30.695, *P* > 0.05), and the relative error between the predicted value and the actual value was small, which all proved the model was practical.

**Conclusion:**

ARIMA (1, 1, 1) can effectively simulate the short-term incidence trend of ILI in Wuhan.

## 1. Introduction

Influenza is an acute respiratory infectious disease caused by influenza virus and the first epidemic to be monitored worldwide [1]. It is mainly transmitted through droplets, and the population is found to be generally susceptible. Influenza is prone to outbreaks or epidemics; on a global scale, the annual incidence of influenza among adults and children is about 5% and 20%, respectively, and the number of death cases associated with seasonal influenza is about 290,000 to 650,000, thus resulting in a huge disease burden [2].

Through influenza surveillance and epidemic early warning, the epidemic trend of influenza can be grasped in time, and scientific support for influenza prevention and control can be provided, which is of great public health significance [3, 4]. At present, there are many methods applied to infectious disease prediction, such as infectious disease dynamic model [5], neural network prediction model [6], grey prediction model [7], logistic regression model [8], and autoregressive integrated moving average model (ARIMA) [9], each with its own advantages and disadvantages.

Among them, the ARIMA model can capture the periodicity, tendency, and randomness of data with high prediction accuracy, and it has been widely used in the prediction of infectious diseases [10–12]. In our study, we predict and verify the incidence of ILI in 2021 by using the ARIMA model to simulate and fit the ILI data extracted from 2014 to 2020 in Wuhan, so as to provide scientific evidence for influenza prevention and control.

The article "Prediction of Incidence Trend of Influenza-Like Illness in Wuhan Based on ARIMA Model" was retracted in 2023. Reasons: signs of a paper mill; suspected computer-generated content; unreliable results or conclusions; lack of ethics approval or compliance.

## 2. Materials and Methods

### 2.1. Data Collection

The data of weekly influenza cases published on the website of China National Influenza Center for influenza surveillance by two sentinel hospitals (Wuhan No. 1 Hospital and Wuhan Children's Hospital) in Wuhan during 2014-2021 were collected, and accordingly, a statistical analysis database was established.

### 2.2. Methods

ARIMA modeling involves three key steps: model identification, parameter estimation, and model diagnosis. Firstly, we determine the applicability of distinguishing weekly ILI cases' incidence by examining stationarity and seasonality and then choose a seasonal ARIMA model if the data shows seasonality. Lastly, according to the results apparently demonstrating the incidence of ILI cases has obvious seasonal characteristics and belongs to time series data, the ARIMA model was proved the best method for the prediction effect analysis of influenza incidence data used in our study.

### 2.3. Statistical Analysis

The data were entered by Excel 2019, and the time series ARIMA model was established and analyzed by SPSS 26.0. At first, the incidence rate of ILI cases is calculated weekly. The prerequisite for ARIMA modeling is stationarity [13]. If the series of weekly incidence rate was found nonstationary while application, the difference and/or data conversion process should be used to process it into a stationary time series. Second, in order to use the ARIMA model method for prediction and analysis, we adopted the form of ARIMA (*P*, *D*, *Q*), where *D* represented the difference order, *P* represented the autoregressive order, and *Q* represents the moving average order. The values of *P* and *Q* came from the autocorrelation function (ACF) diagram and partial autocorrelation function (PACF) diagram made by stationary series. Third, the least square method was used to estimate the parameters of the selected model and the significance of the statistic Ljung-Box *Q* was tested. Fourth, goodness of fit test and white noise test were used to judge the fitting effect of the model, and parameter independence test was used to judge the independence and randomness of ACF and PACF. Finally, we fit the weekly ILI data of Wuhan in 2021 according to the best established ARIMA model and compared it with the actual incidence aim to evaluate the prediction effect of the model.

## 3. Results

### 3.1. Sequence Stabilization

The time series diagram of weekly ILI in Wuhan from 2014 to 2020 was drawn (Figure 1). It can be seen from the graph that the sequence of ILI was nonstationary, and the overall trend was fluctuated. The incidence after 2018 fell, while in the spring of 2020 it was high and then fell later. In order to meet the preconditions for establishing the stability of model modeling, the heteroscedasticity of data series was eliminated, and the original data was differentiated to eliminate the influence. In consideration of the loss of original data due to the difference, the number of difference orders should be minimized. After the first-order difference of the original sequence, the sequence basically tended to be stable and the graph was good (Figure 2), so the difference order *D* = 1.

The article "Prediction of Incidence Trend of Influenza-Like Illness in Wuhan Based on ARIMA Model" was retracted in 2023. Reasons: signs of a paper mill; suspected computer-generated content; unreliable results or conclusions; lack of ethics approval or compliance.

### 3.2. Model Identification

We calculated the autoregressive order *P* and moving average order *Q* through model identification. First, we draw the first-order difference sequence ACF and PACF and observe whether the statistics have significant differences to rank *P* and *Q*. ACF showed the property of truncation (Figure 3). When PACF lag = 3, it showed truncation, but *P* and *Q* generally did not exceed 2 (Figure 4). According to the order determination standard, the *P* value was determined to be 1 or 2, and the *Q* value was 1 or 2. Combined with the *D* value, it was preliminarily determined that the models to be selected are ARIMA (1, 1, 1), ARIMA (1, 1, 2), ARIMA (2, 1, 1), or ARIMA (2, 1, 2).

### 3.3. Model Diagnosis

Parameter estimation and Ljung-Box *Q* statistic test were carried out for the alternative model, and goodness of fit and residual test were also further carried out. Akaike information criterion (AIC) and Schwarz Bayesian criterion (SBC) were used to judge the fitting effect. The standard was that the smaller the value of AIC and SBC, the better the fitting effect. In this study, the AIC and SBC values of the ARIMA (1, 1, 1) model were the smallest among the four models (Table 1), which exhibited that the ARIMA (1, 1, 1) model was proven as the most optimal one. Moreover, through the autocorrelation diagram we made for its residual sequence (Figure 5), both ACF and PCAF did not exceed 95% confidence interval, suggesting that the residual was independently distributed. Ljung-Box *Q* statistics had no statistical significance (*P* > 0.05), and its minimum value was 0.018, *P* = 0.893, while the maximum value was 30.695, *P* = 0.719, which accurately reflected the residual conformed to the white noise sequence. In conclusion, the ARIMA (1, 1, 1) model can be considered as the best model with its proper fitting.

### 3.4. Model Evaluation

The established ARIMA (1, 1, 1) model was used to predict the annual ILI data of Wuhan City in 2021, and the fitting effect diagram between the predicted value and the actual value was drawn (Figure 6). On the whole, the overall trend of the prediction results of the model is basically consistent with the actual situation, and the relative error was small, indicating that the model can better simulate the incidence of influenza in this period. The incidence prediction results for the 52 weeks of year 2021 showed that the measured values in the second week exceeded the 95% confidence interval, and other weeks were all within the 95% confidence interval (Table 2).

The article "Prediction of Incidence Trend of Influenza-Like Illness in Wuhan Based on ARIMA Model" was retracted in 2023. Reasons: signs of a paper mill; suspected computer-generated content; unreliable results or conclusions; lack of ethics approval or compliance.

## 4. Discussion

Influenza is closely related to each of us. As reported in previous studies, influenza virus is very prone to mutation, which will lead to influenza pandemic every year and result in huge social burden and medical consumption. As a country with a large population, China has implemented many prevention policies against influenza and established relevant health supervision systems; however, influenza is still prevalent in China. There are many factors affecting the incidence rate of influenza, including population mobility, environment, virus virulence, geographical location, prevention strategies, and economic status [14]. When the population base changes little, the corresponding dynamic model can be established according to the change law of the time series of ILI, which can effectively predict the influenza epidemic. In this study, we introduced the statistical method of the ARIMA model to construct and predict the incidence rate of influenza, so as to provide research ideas for influenza prevention and public health guidance.

Epidemiological monitoring of infectious diseases is very common, and model prediction can make better use of monitoring data. Researches have proved that the statistical model is helpful to predict the incidence rate of infectious diseases, which is very important for the health sector to identify the spread of epidemics as soon as possible. The autoregressive moving average hybrid model of time series analysis was originally designed for economics [15, 16]. However, it played an important role in the prediction of infectious diseases (influenza, malaria, varicella, and others) and had been widely used at present. The ARIMA model can accurately forecast the occurrence of future disease through weekly, monthly, or annual incidence rate data [17, 18], and with its characteristics of simplicity and good short-term prediction effect, it has become one of the most commonly used time series models in the field of infectious diseases.

Based on the data of influenza-like cases in Wuhan, this study constructed a weekly influenza incidence rate model from 2014 to 2020 using ARIMA. Then, we used the model to predict the weekly incidence rate of influenza in 2021 and compared the predicted value with the actual value; as a result, the overall trend of the two groups of data was found basically the same, which indicated that the ARIMA model has good prediction ability and can make a reasonable prediction for the future trend based on the previous data. Therefore, the ARIMA (1, 1, 1) model was very effective in predicting the incidence rate of influenza in Wuhan, which provided a basis for early warning analysis in the future. When the predicted incidence rate increases significantly, we can take relevant policies or improvement measures in advance, such as health publicity, personal protection, and vaccination, so as to reduce the loss as much as possible.

The article "Prediction of Incidence Trend of Influenza-Like Illness in Wuhan Based on ARIMA Model" was retracted in 2023. Reasons: signs of a paper mill; suspected computer-generated content; unreliable results or conclusions; lack of ethics approval or compliance.

Nowadays is the era of big data, and a large amount of data is penetrating into all aspects of our daily life. Taking full advantage of data in public health is of great importance for disease warning [19, 20]. Time series analysis of incidence rate data is helpful to put forward new hypotheses, predict epidemic trends, and improve the prevention and control system. In our study, the ARIMA model is constructed to predict the incidence rate of influenza, provide reference for the influenza early warning system, and help public health decision-makers adopt preventive and control measures in time to reduce medical consumption and social burden. At the same time, our research also has some limitations. For example, the ARIMA model is only suitable for short-term prediction and infectious diseases have their complexity. Thus, continuous monitoring is very necessary [21]. In the future, we will establish a dynamic adjustment model through further model improvement and more reliable influenza data, so as to provide a more sufficient scientific basis for influenza epidemic prevention and control.

## Figures and Tables

**Figure 1:** Time series of incidence rate of influenza from 2014 to 2020.

**Figure 2:** Time series diagram of influenza incidence rate after first-order difference.

**Figure 3:** Autocorrelation chart of influenza incidence rate from 2014 to 2020 after first-order difference.

**Figure 4:** Partial autocorrelation chart of influenza incidence rate from 2014 to 2020 after first-order difference.

**Figure 5:** Residual autocorrelation diagram and partial autocorrelation diagram.

**Figure 6:** Forecast of incidence rate of influenza from 2014 to 2021.

**Table 1:** Goodness of fit test of the model to be selected.

Statistic	Model to be selected			
	ARIMA (1, 1, 1)	ARIMA (1, 1, 2)	ARIMA (2, 1, 1)	ARIMA (2, 1, 2)
Standard error	0.792	0.796	0.797	0.797
Log likelihood	-429.464	-430.899	-431.233	-430.851
AIC	862.929	867.798	868.466	869.703
SBC	870.718	879.481	880.149	885.281

Note: AIC: Akaike information criterion; SBC: Schwarz Bayesian criterion.

The article "Prediction of Incidence Trend of Influenza-Like Illness in Wuhan Based on ARIMA Model" was retracted in 2023. Reasons: signs of a paper mill; suspected computer-generated content; unreliable results or conclusions; lack of ethics approval or compliance.

**Table 2:** Comparison between actual and predicted ILI in 52 weeks of year 2021.

Week	Actual incidence rate	Predicted incidence rate	Predicted incidence rate 95% CI		Week	Actual incidence rate	Predicted incidence rate	Predicted incidence rate 95% CI	
			Lower limit	Upper limit				Lower limit	Upper limit
1	2.17	1.01	-0.54	2.56	27	0.14	0.99	-2.59	4.58
2	4.55	1.03	-1.05	3.12	28	0.08	0.98	-2.6	4.57
3	0.41	1.05	-1.38	3.48	29	0.10	0.97	-2.61	4.56
4	0.37	1.06	-1.62	3.75	30	0.07	0.96	-2.62	4.55
5	0.38	1.07	-1.8	3.95	31	0.10	0.95	-2.64	4.54
6	0.03	1.08	-1.93	4.1	32	0.08	0.94	-2.65	4.53
7	0.19	1.09	-2.04	4.22	33	0.08	0.93	-2.66	4.52
8	0.19	1.09	-2.12	4.31	34	0.07	0.92	-2.67	4.51
9	0.05	1.1	-2.19	4.38	35	0.19	0.91	-2.68	4.5
10	0.07	1.1	-2.25	4.44	36	0.14	0.9	-2.69	4.49
11	0.20	1.1	-2.29	4.48	37	0.29	0.89	-2.71	4.48
12	0.26	1.1	-2.33	4.52	38	0.32	0.88	-2.72	4.47
13	0.16	1.09	-2.36	4.55	39	0.40	0.87	-2.73	4.46
14	0.33	1.09	-2.39	4.57	40	0.18	0.85	-2.74	4.45
15	0.26	1.09	-2.41	4.58	41	0.33	0.84	-2.75	4.44
16	0.21	1.08	-2.43	4.59	42	0.21	0.83	-2.76	4.43
17	0.21	1.07	-2.45	4.6	43	0.29	0.82	-2.77	4.41
18	0.25	1.07	-2.47	4.61	44	0.21	0.81	-2.79	4.4
19	0.24	1.06	-2.49	4.61	45	0.15	0.8	-2.8	4.39
20	0.31	1.05	-2.5	4.61	46	0.19	0.79	-2.81	4.38
21	0.14	1.05	-2.51	4.61	47	0.15	0.77	-2.82	4.37
22	0.12	1.04	-2.53	4.6	48	0.27	0.76	-2.83	4.36
23	0.15	1.03	-2.54	4.6	49	0.28	0.75	-2.84	4.35
24	0.16	1.02	-2.55	4.6	50	0.38	0.74	-2.86	4.34
25	0.08	1.01	-2.57	4.59	51	0.48	0.73	-2.87	4.32
26	0.05	1	-2.58	4.58	52	0.81	0.72	-2.88	4.31

## Data Availability

The datasets used and analyzed during the current study are available from the corresponding author upon reasonable request.
